The article "COVID-19 knowledge, attitude, and preventive practices among government and private bank workers in Ethiopia" was retracted in 2026. Reason: duplicate publication.

# COVID-19 knowledge, attitude, and preventive practices among government and private bank workers in Ethiopia

**DOI:** 10.3389/fpubh.2023.1251701

**Published:** 2023-10-30

**Authors:** Seada Hassen, Metadel Adane

**Affiliations:** Department of Environmental Health, College of Medicine and Health Science, Wollo University, Dessie, Ethiopia

**Keywords:** bank workers, COVID19, knowledge, attitude, preventive practice, Ethiopia

## Abstract

**Background:**

Bank workers are among the many service-sector employees who are at risk of COVID-19 infection. Individual’s adherence to control measures is affected by their COVID-19 knowledge, attitudes, and practices (KAP). Since KAP is an important cognitive key in public health prevention and promotion, this study aimed to identify COVID-19 KAP-related gaps among bank workers in Dessie City, Ethiopia and to guide banks and health authorities in taking corrective actions.

**Methods:**

An institution-based cross-sectional study was conducted from January 1st to 30th, 2021 among 413 bank workers. A binary logistic regression was applied to determine association of independent variables with outcome variables using three different models. Variables at 95% confidence interval (CI) with a *p* < 0.25 from bivariate analysis were transported to three different multivariable logistic regression models and then variables with a *p-*value of 0.05 from the multivariable analysis of each model were declared as significantly associated with the outcome variables.

**Results:**

The results of this study show that 84.7% [95% CI: 81.1–88.1] of bank workers had good knowledge, 50.4% positive attitude, and 50.6% [95% CI: 45.8–55.0] good practice towards prevention of COVID-19. The only variable significantly associated with knowledge in this study was positive attitude (AOR = 8.89; 95%CI: 3.34–23.64). Being ≥35 years old (AOR = 2.46; 95%CI: 1.25–4.84) and getting information on COVID-19 (AOR = 3.81; 95%CI: 1.84–7.91) were among factors significantly associated with attitude towards COVID-19 prevention, whereas being female and ≥ 35 years old (AOR = 2.56; 95%CI: 1.29–5.06) and (AOR = 2.73; 95% CI: 1.15–6.51), respectively were factors associated with good preventive practice towards COVID-19.

**Conclusion and recommendation:**

Considering those significant factors responsible for determining COVID-19 KAP level of respondents, health education program and information dissemination are recommended, including appropriate strategies by policy makers and bank managers to develop effective interventions for COVID-19 transmission in banks.

## Background

Coronaviruses are a group of viral pathogens, some of which can cause illnesses predominantly in the human respiratory tract, and also in the gastrointestinal, hepatic, and cardiovascular systems (1). Outbreaks of coronavirus infections in earlier years include the Middle East respiratory syndrome (MERS) and severe acute respiratory syndrome (SARS), both of which posed a major public health concern (2, 3). Coronavirus disease 2019 (COVID-19) is an emerging respiratory disease that was first reported in Wuhan, Hubei state, China, on 31 December 2019 as a cluster of pneumonia cases. The responsible pathogen for the disease is severe acute respiratory syndrome coronavirus 2 (SARS-CoV-2) (1, 4–6). The WHO report on 2021 showed more than 160 million confirmed COVID-19 cases and 3.3 million deaths (7).

The causative agent for this infection was confirmed as a novel coronavirus on 7 January 2020. WHO declared that the outbreak of COVD-19 was characterized as international public health emergency on January 30, 2020, and as a pandemic on 11 March 2020 (8). SARS-CoV-2 virus is the seventh known coronavirus to infect humans (9–12). COVID-19 has an average incubation period of 5 days with a range between 2 and 14 days (13, 14), and it shows a mild course in 80% of observed cases and a severe course in 20%, with a lethality rate of 0.3–5.8% (15). Distinctive symptoms that are common in COVID-19 patients are fever, dry cough, sore throat, myalgia, fatigue, and shortness of breath (1, 16, 17).

On February 14, 2020, the first case of COVID-19 was recorded on the African continent (18). In Ethiopia, on 13th of March 2020, the Federal Ministry of Health confirmed and reported the first imported case of COVID-19 in Addis Ababa, Ethiopia (19–21). Highly communicable nature of COVID-19 pandemic attributed the response of the infection in Ethiopia harsher and dangerous. Besides, a very swift transmission of viruses distributed within 213 countries, including Ethiopia. From this study KAP’s practices are inadequate to fight and minimize the impacts of the pandemic in Ethiopia (22). COVID-19 vaccines were developed (23) and tested by late 2020, hence the most practical way for many communities to reduce the chance of COVID-19 transmission is to implement reliable protection and precaution strategies (17, 24).

Ethiopian bank workers are among the many service-sector employees who have frequent and close interaction with many people (25, 26) and retail banking in Ethiopia, both of which allow the chance of COVID-19 exposure to spread among various individuals (27). Therefore, applying preventive measures is mandatory among bank workers (28). People’s adherence to control measures is affected by their COVID-19 knowledge, attitudes, and practices (29, 30). KAP is an important cognitive key in public health prevention and promotion. It involves a range of beliefs about the causes of the disease and exacerbating factors, identification of symptoms, and available methods of treatments and consequences (31). And also, KAP of people towards COVID-19 disease help in determining a community’s readiness to accept behavioral change measures, while understanding these factors may guide strategies to strengthen the effectiveness, compliance with and success of infection prevention and control measures adopted in a country (32).

Assessing the KAP of bank workers associated with COVID-19 preventative measures is necessary to determine where gaps are and to guide corrective steps. Therefore, the goal of this study was to determine the KAP toward COVID-19 among bank employees in Dessie, Ethiopia.

## Materials and methods

### Study area description

This research was carried out in banks found in Dessie, a city in the South Wollo Zone, located in the eastern part of Amhara state in north-central Ethiopia, 401 kilometers from the country’s capital, Addis Ababa. Dessie City had a total population of 151,174 people as estimated in the national census conducted by Ethiopia’s Central Statistical Agency (CSA) in 2007, including 72,932 males and 78,242 females. An estimate in 2019 show the number of bank branches in Dessie city was 41, including 17 government and 24 private bank branches employing a total of 2,647 employees. The majority of the city’s bank branches are commercial bank branches (33, 34).

### Study design, population, and study period

An institution-based cross-sectional study was performed among bank employees in Dessie City from January 1st to 30th, 2021. The source population consisted of all workers in Dessie City bank branches, whereas the study population consisted of chosen bank workers from Dessie City bank branches.

### Sample size determination and sampling procedure

Single population proportion formula was used to determine the sample size considering the assumptions that the proportion of KAP in institutions including banks of Dessie City as 50% (since there had been no previous study conducted on bank workers in the study area so far), a 95% CI and 5% margin of error (35). After considering a 10% non-response rate from the initial calculated sample size, the final sample size for this study became 422.

Dessie City has a total of 41 bank branches, including 17 government and 24 private bank branches, of which 50% (21 bank branches) were selected randomly to be included in this study. The number of bank employees to be included was taken using salary documents (payroll) from each branch. Employees on the branch payroll list were picked at random from the payroll document by proportionally assigning the entire sample to the total number of workers in the selected bank branches.

### Operational definition

#### Bank workers

Both back and frontline bank officials in charge of taking client cash deposits, utility payments, documenting transactions, printing receipts, cashing checks, and counseling customers on investments, foreign currency exchange, and loans. They are frequently in contact with consumers every day (27).

#### Good or poor knowledge

Bank workers who correctly responded correctly to more than or equal to the mean of 16 knowledge questions (Table 1) were deemed to have good knowledge about COVID-19, while those who replied correctly less than the mean value were considered to have poor knowledge (36).

**Table 1:** Knowledge about COVID-19 among bank workers in Dessie City, Ethiopia, January 2021.

Knowledge question	Yes	No
	*n* (*%*)	*n* (*%*)
COVID-19 is caused by virus.	398 (96.4)	15 (3.6)
The signs and symptoms of COVID-19 include fever, fatigue, dry cough and shortness of breath.	377 (91.3)	36 (8.7)
Unlike the common cold, stuffy nose, runny nose, and sneezing are less common in persons infected with the COVID-19 virus.	383 (92.7)	30 (7.3)
Currently there is no vaccine available for COVID-19 in Ethiopia.	383 (92.7)	30 (7.3)
There is no effective curative treatment for COVID-19.	391 (94.7)	22 (5.3)
Only those who are older or have underlying disease are at a high risk of deterioration into serious condition as a result of COVID-19.	380 (92.0)	33 (8.0)
The main mode of COVID-19 transmission is through contact only.	383 (92.7)	30 (7.3)
People without symptoms can still transmit COVID-19 to others.	386 (93.5)	27 (6.5)
Persons with COVID-19 cannot infect/spread the virus to others when a fever is not present.	384 (93.0)	29 (7.0)
Eating or having contact with wild animals would result in the infection by the COVID-19 virus.	394 (95.4)	19 (4.6)
The time from exposure to onset of symptoms is 2–14 days.	383 (92.7)	30 (7.3)
Mask wearing prevents infection by the COVID-19 virus.	384 (93.0)	29 (7.0)
Isolation and treatment of people who are infected with the COVID-19 virus are effective ways to reduce the spread of the virus.	387 (93.7)	26 (6.3)
Proper washing of hands for at least 20 s with soap and water is one method of preventing COVID-19.	390 (94.4)	23 (5.6)
There is a need to wash hands before and after touching all things outside your home.	381 (92.3)	32 (7.7)
Being 2 meters apart from individuals can reduce the risk of transmission of COVID-19.	396 (95.9)	17 (4.1)

Mean ± standard deviation = 14.96 ± 2.81; minimum = 0 and maximum = 16.

#### Positive or negative attitude

Those bank employees responding positively to more than or equal to the mean out of 11 attitude questions (Table 2) were considered as having a positive attitude towards taking precautions to prevent COVID-19 transmission, while those who answered positively to less than the mean were judged to have negative attitude (37).

**Table 2:** Attitude toward COVID-19 precautions among bank workers in Dessie City, Ethiopia, January 2021.

Attitude question	Agree	Neutral	Disagree
	*n* (%)	*n* (%)	*n* (%)
COVID-19 is a serious disease.	380 (92.0)	7 (1.7)	26 (6.3)
Wearing a well-fitting face mask is effective in preventing COVID-19 virus transmission.	382 (92.5)	14 (3.4)	17 (4.1)
Hand washing can protect you from COVID-19 virus.	384 (92.9)	27 (6.5)	2 (0.5)
COVID 19 is not stigmatized and I should not hide my infection.	223 (54.0)	13 (3.1)	177 (42.9)
Self-efficacies are mandatory to control COVID-19.	255 (61.8)	17 (4.1)	141 (34.2)
I believe I can protect myself against COVID-19.	229 (55.5)	29 (7.0)	155 (37.6)
There is personal risk of being infected (vulnerability) with COVID-19 while in crowded place and meeting with many people.	262 (63.5)	101 (24.5)	50 (12.1)
I will not go to hospital even if I get sick because of the risk of getting infected with COVID-19.	71 (17.2)	81 (19.6)	261 (63.2)
COVID-19 can eventually be successfully controlled.	229 (55.5)	133 (32.2)	51 (12.3)
If there is an available lab test for detection of the virus, I am willing to do it.	308 (74.6)	70 (16.9)	35 (8.5)
If there is an available vaccine for the virus, I am willing to get it.	166 (40.2)	96 (23.2)	151 (36.6)

Mean ± standard deviation = 39.54 ± 7.78; Minimum = 20 and maximum = 55.

#### Good or poor practice

Bank employees who responded positively to more than or equal to the mean out of seven practice questions (Table 3) were considered as having good practice to prevent COVID-19 transmission, while those who answered positively to less than the mean were considered to have poor practice (37).

**Table 3:** Practice of COVID-19 preventive measures among bank workers in Dessie City, Ethiopia, January 2021.

Practice question	Always	Sometimes	Never
	*n* (*%*)	*n* (*%*)	*n* (*%*)
Go out less often to crowded places and maintain an appropriate social distance from others.	68 (16.5)	171 (41.4)	174 (42.1)
Wear a face mask when leaving home to go to work place or other crowded area.	144 (34.9)	256 (62.0)	13 (3.1)
Perform hand hygiene before putting on and after removing a mask.	112 (27.1)	149 (36.1)	152 (36.8)
Wash hands with liquid soap and water and rub for at least 20 s.	120 (29.1)	283 (68.5)	10 (2.4)
Perform hand hygiene with 70–80% alcohol-based hand rub if hand washing facilities are not available.	98 (23.7)	268 (64.9)	47 (11.4)
Avoid touching animals, poultry/birds or their droppings.	301 (72.9)	81 (19.6)	31 (7.5)
Follow the updates about the spread of the virus.	154 (37.3)	250 (60.5)	9 (2.2)

Mean ± standard deviation = 15.36 ± 2.92; Minimum = 7 and maximum = 21.

### Data collection procedures and quality assurance

Using a WHO report on COVID-19 (38), an Ethiopian Ministry of Health report (39) and a study of various literature to ensure their validity (28, 29, 40, 41), a structured questionnaire and an observational checklist were constructed. The questionnaire was created in English, translated into Amharic, and then retranslated to English to maintain uniformity of questions.

The questionnaire included questions on socio-demographics, knowledge, attitude, and practice, as well as medical history and source of COVID-19 information. The questionnaire had a total of 16 questions to assess COVID-19 knowledge. Knowledge about signs and symptoms, transmission channels, as well as prevention and control were all included in the questions. One point was given for each question that was correctly answered, while zero points were given for each item that was erroneously answered or left unanswered by selecting the response “do not know.” The prospective knowledge scores ranged from 0 to 16, with a score higher than the mean indicating that the person knew more about COVID-19 than the average bank worker (29).

Attitudes towards COVID-19 prevention were assessed using 11 questions that covered two aspects of attitude: the participants’ perceived risk of disease and their perceived self-efficacy in controlling the disease. Each item’s response on attitude towards taking precautions against COVID-19 was categorized measured on a scale of 5 ranging from 1 (strongly disagree) to 5 (strongly agree). The mean score of each subscale was calculated to indicate the degrees of participant’s attitudes in the respective domains (14).

Personal cleanliness, facemask usage, and maintaining social distance were among the seven questions used to assess COVID-19 prevention strategies used and each response was measured on a scale of 3: 1 (never), 2 (sometimes), and 3 (always). A higher score showed that the preventative measures were being implemented to a higher degree (14).

The questionnaire was pretested on five bank branches (3 governments and 2 private) that accounted for 5% of the total sample size and had not been selected for the research before the real data collecting began. The information was gathered through self-administered questionnaire that included socio-demographic, knowledge and attitude questions, while preventive strategies and equipment used to apply preventive measures were determined by observation.

Three data collectors having environmental health background were recruited and given 1 day of training on the study’s objectives, data collecting instruments, and ethical issues; they distributed the questionnaire for self-administered data collection and used the checklist to observe the preventive strategies-related questions in the bank environment. On a daily basis, the investigator and supervisors verified the questionnaires for completeness and data quality control. To guarantee the questionnaire’s reliability, data input was re-checked in a randomly selected 10% of the surveys and data cleaning was also performed prior to statistical analysis.

### Data management and analysis

Before being exported to Statistical Package of the Social Science (SPSS) version 25.0 for analysis, data was verified for completeness, coded, and entered into Epi-Data version 4.6. To examine the distribution of data, descriptive analysis was presented using frequencies with percentages (%) for categorical variables and mean with standard deviations (SD) for continuous variables.

Binary logistic regression [crude odds ratio (COR)] was applied to determine association of independent variables with COVID-19 knowledge, attitude or preventive practice at 95% confidence interval (CI). Variables with *p* < 0.25 were transported to three different multivariable logistic regression [adjusted odds ratio (AOR)] models to identify factors independently associated with knowledge, attitude or preventive practice at a 95% CI to see the strength and significance of the association. In the first model, factors significantly associated with good knowledge about COVID-19 were identified; in the second model, factors significantly associated with positive attitudes towards taking precautionary measures for COVID-19 were identified; and in the third model, factors significantly associated with good COVID-19 preventive practices were identified. Multicollinearity testing was carried out between independent variables where the standard error cut-off point was found to be greater than 2 for all independent variables in the three models. The Hosmer and Lemeshow goodness-of-fit test was applied to the three models; we found a *p*-value of 0.875, 0.935, and 0.897 for Model I, Model II, and Model III, respectively, indicating that the all models were fit.

### Ethics approval and consent to participate

All study methods were performed in accordance with the ethical principles of the Declaration of Helsinki (42). This study received ethical approval from Wollo University College of Medicine and Health Science’s Ethical Review Committee, with ethical review reference number CMHS145/02/13. Letters of authorization from government and commercial bank branches, as well as the Dessie City health department were secured. Data collectors were advised to wear facemasks, use hand sanitizer, and keep a physical distance of two meters when distributing and collecting surveys from bank workers, as per WHO standards.

Before starting the interviews, the data collectors explained the purpose of the study to all the participants and written informed consent was given obtained from study participants prior to the start of data collection. The confidentiality and anonymity of the study participants’ related data were maintained by avoiding possible identifiers such as participants’ names. Identification code numbers only were used as a reference. Employees of the bank who were not wearing a facemask at the time of the interview were strongly advised to do so.

## Results

### Socio-demographic and economic characteristics of bank workers

The response rate from the total sample of 422 was 413 (97.9%) in this study. Data were collected from 208 (50.4%) government and 205 (49.6%) private bank branches. A majority of respondents 225 (54.5%) were Orthodox Christians, over one-third Muslims 162 (39.2%), 24 (5.8%) Protestants and 2 (0.5%) Catholics; those of Amhara ethnicity numbered 357 (86.4%) and the remaining were 42 (10.2%) Oromo, and 14 (3.4%) Tigre. Of the total respondents, 312 (75.5%) were urban residents (Table 4).

**Table 4:** Socio-demographic, economic, medical history-related and source of COVID-19 information-related factors on COVID-19 KAP among bank workers in Dessie City, Ethiopia, January 2021.

Variable	Category	Frequency (*n*)	Percentage (*%*)
Bank branch	Government	208	50.04
	Private	205	49.6
Sex of respondent	Male	233	56.4
	Female	180	43.6
Age of respondent (years)	18–34	247	59.8
	≥35	166	40.2
Education level	Diploma	101	24.5
	1st degree	180	43.6
	2nd degree	132	32.0
Monthly income (dollar)	110.74–259.16	210	50.8
	259.17–598.00	203	49.2
Marital status	Not married	179	43.3
	Married	234	56.7
Experience in the bank (years)	<2	71	17.2
	2–5	194	47.0
	>5	148	35.8
Position as cashier (days per week)	0–4	130	31.5
	5–6	283	68.5
Family size (persons)	<5	245	59.3
	≥5	168	40.7
Have children	No	196	47.5
	Yes	217	52.5
Have family member >65 years	No	333	80.6
	Yes	80	19.4
Presence of respiratory conditions	No	301	72
	Yes	112	27.1
Presence of chronic illness	No	333	80.6
	Yes	80	19.4
Presence of poster showing COVID-19 preventive measures in workplace	No	322	78.0
	Yes	91	22.0
Received training on COVID-19	No	309	74.8
	Yes	104	25.2
Received health information on COVID-19	No	95	23.0
	Yes	318	77.0

Mean work experience ± standard deviation = 5.56 ± 3.65; minimum = 1 and maximum = 22. 1, reference category; COR, crude odds ratio; CI, confidence interval.

### Medical history-related and source of COVID-19 information factors

A majority of the bank workers [301 (72.9%) and 333 (80.6%)] had no respiratory or chronic illness, respectively. From the total of 318 (77%) bank workers who had received health information about COVID-19, 62.2% had received the health information from television, 51.6% from radio and newspaper, 38.5% from social media, and 27.1% from friends and healthcare providers (Table 4).

### Proportion of knowledge about COVID-19 and associated factors

More than three-fourths of the bank workers (84.7% [95% CI: 81.1–88.1]) had good knowledge about COVID-19 while 15.3% (95% CI: 11.9–18.9) had poor knowledge. Almost all 398 (96.4%) of bank workers knew that COVID-19 is a viral diseases and 377 (91.3%) of them knew the major signs and symptoms of COVID-19 include fever, fatigue, dry cough and shortness of breath (Table 1).

Multivariable analysis from the model for COVID-19 knowledge showed that only attitude towards taking COVID-19 precautions was significantly associated with knowledge about COVID-19. A main finding of the study shows that those having a positive attitude towards taking COVID-19 precautions were 8.89 times more likely to have good knowledge about COVID-19 than those who had a negative attitude (Table 5).

**Table 5:** Factors associated with knowledge about COVID-19 among bank workers in Dessie City, Ethiopia, January 2021.

Variable	Category	Knowledge level				
		Good	Poor	COR (95% CI)	AOR (95% CI)	*p*-value
Sex of respondent	Male	193	40	1	1	
	Female	157	23	1.42 (0.81–2.46)	0.72 (0.37–1.39)	0.328
Age of respondent (years)	18–34	196	51	1	1	
	≥35	154	12	3.34 (1.72–6.48)	0.85 (0.32–2.28)	0.747
Education level	Diploma	85	16	1	1	
	1st degree	143	37	0.73 (0.38–1.39)	0.54 (0.26–1.14)	0.108
	Masters	122	10	2.30 (0.99–5.31)	0.78 (0.21–2.91)	0.708
Monthly income (dollar)	110.74–259.16	166	44	1	1	
	259.17–598.00	184	19	2.57 (1.44–4.57)	1.17 (0.45–3.03)	0.744
Marital status	Not married	138	41	1	1	
	Married	212	22	2.86 (1.63–5.02)	1.37 (0.68–2.78)	0.381
Experience in the bank (years)	<2	56	15	1	1	
	2–5	155	39	1.07 (0.55–2.08)	1.07 (0.51–2.26)	0.858
	>5	139	9	4.12 (1.71–10.0)	1.23 (0.36–4.24)	0.742
Family size (persons)	<5	194	51	1	1	
	≥5	156	12	3.42 (1.76–6.63)	1.12 (0.47–2.67)	0.798
Have children in household	No	154	42	1	1	
	Yes	196	21	2.55 (1.45–4.48)	1.25 (0.62–2.51)	0.535
Presence of poster showing COVID-19 preventive measures at work	No	266	56	1	1	
	Yes	84	7	2.53 (1.11–5.75)	1.99 (0.81–4.93)	0.135
Received training on COVID-19	No	255	54	1	1	
	Yes	95	9	2.23 (1.06–4.70)	1.02 (0.40–2.61)	0.966
Received health information on COVID-19	No	68	27	1	1	
	Yes	282	36	3.11 (1.77–5.47)	1.44 (0.74–2.81)	0.281
Attitude toward COVID-19 prevention measures	Negative	148	57	1	1	
	Positive	202	6	12.97(5.45–30.87)	8.89 (3.34–23.64)	<0.001*

AOR, adjusted odds ratio; COR, crude odds ratio; CI, confidence interval; 1, reference category. *Significant association.

### Proportion of attitude about COVID-19 and associated factors

Half of the bank workers (50.4% [95% CI: 45.5–55.0]) had a positive attitude towards taking precautions against COVID-19. A majority of the bank workers (92%) agreed that COVID-19 is a serious disease. In relation to precautionary measures taken to prevent COVID-19, a majority of the bank workers (92.5 and 92.9%) agreed that wearing a well-fitting face mask and hand washing, respectively, are effective in preventing COVID-19 disease (Table 2).

Multivariable analysis from the attitude model revealed that those 35 years of age or over were 2.46 times more likely to have a positive attitude towards taking precautions for COVID-19 than those who were 18–34, married bank workers were 2.51 times more likely have a positive attitude towards taking COVID-19 precautions than those who were unmarried, and those individuals who had children were 1.95 times more likely to have a positive attitude towards taking COVID-19 precautions than those who did not have children. Furthermore, bank workers who had received health information about COVID-19 were 3.81 times more likely to have a positive attitude towards taking COVID-19 precautions than those who had not received such information. Additionally, those bank workers who had good knowledge about COVID-19 were 10.22 times more likely to have a positive attitude towards taking precaution against COVID-19 than those who had poor knowledge about COVID-19 (Table 6).

**Table 6:** Factors associated with attitude about COVID-19 among bank workers in Dessie City, Ethiopia, January 2021.

Variable	Category	Attitude level				
		Positive	Negative	COR (95%CI)	AOR (95%CI)	*p*-value
Sex of respondent	Male	96	137	1	1	
	Female	112	68	2.35 (1.58–3.50)	1.37 (0.81–2.32)	0.240
Age of respondent (years)	18–34	79	168	1	1	
	≥35	129	37	7.41 (4.71–11.66)	2.46 (1.25–4.84)	0.009*
Education level	Diploma	38	63	1	1	
	1st degree	75	105	1.18 (0.72–1.95)	0.56 (0.27–1.17)	0.125
	2nd degree	95	37	4.26 (2.45–7.40)	0.49 (0.17–1.45)	0.195
Monthly income (dollar)	110.74–259.16	69	141	1	1	
	259.17–598.00	139	64	4.44 (2.94–6.71)	1.88 (0.82–4.31)	0.134
Marital status	Not married	49	130	1	1	
	Married	159	75	5.62 (3.67–8.63)	2.51 (1.41–4.45)	0.002*
Experience in the bank	<2 years	24	47	1	1	
	2–5 years	64	130	0.96 (0.54–1.71)	0.68 (0.33–1.39)	0.289
	>5 years	120	28	8.39 (4.42–15.93)	1.84 (0.72–4.67)	0.201
Family size (persons)	<5	86	159	1	1	
	≥5	122	46	4.90 (3.19–7.53)	1.40 (0.79–2.48)	0.247
Have children	No	66	130	1	1	
	Yes	142	75	3.73 (2.48–5.61)	1.95 (1.15–3.32)	0.014*
Presence of poster showing COVID-19 preventive measures at work	No	154	168	1	1	
	Yes	54	37	1.59 (0.99–2.55)	0.87 (0.46–1.64)	0.659
Training on COVID-19	No	132	177	1	1	
	Yes	76	28	3.64 (2.23–5.93)	0.72 (0.34–1.49)	0.371
Have health information on COVID-19	No	18	77	1	1	
	Yes	190	128	6.35 (3.63–11.11)	3.81 (1.84–7.91)	<0.001*
Knowledge about COVID-19	Poor	6	57	1	1	
	Good	202	148	12.97 (5.45–30.87)	10.22 (3.65–28.62)	<0.001*

AOR, adjusted odds ratio; COR, crude odds ratio; CI, confidence interval; 1, reference category. *Significant association.

### Proportion of preventive practice toward COVID-19 and associated factors

Half of the bank workers who participated in this study (50.6% [95% CI: 45.8–55.0]) practiced good COVID-19 preventive measures. Only 68 (16.5%) of the bank workers reported going out less frequently to crowded places and always maintaining an appropriate social distance with others. Around one-third (34.9%) always wore a facemask when leaving home, 29.1% washed their hands with soap and 23.7% used hand sanitizer (Table 3).

From multivariable analysis of the model for bank workers’ practice of COVID-19 preventive measures, we found that females were 2.56 times more likely to have a good practices than males, those 35 years of age or over were 2.73 times more likely to have good practices than those who were 18–34, those bank workers having 2–5 years’ work experience were 0.26 times less likely to have good practice than those who had less than 2 years’ experience. Furthermore, those who had a positive attitude were 35.4 times more likely to practice good COVID-19 preventive measures than those who had a negative attitude (Table 7).

**Table 7:** Factors associated with practice of COVID-19 preventive measures among bank workers in Dessie City, Ethiopia, January 2021.

Variable	Category	Practice level				
		Good	Poor	COR (95% CI)	AOR (95 CI)	*p*-value
Bank branch type	Government	119	89	1.71 (1.16–2.52)	0.87 (0.43–1.75)	0.687
	Private	90	115	1	1	
Sex of respondent	Male	91	142	1	1	
	Female	118	62	2.97 (1.98–4.45)	2.56 (1.29–5.06)	0.007*
Age of respondent (years)	18–34	78	169	1	1	
	≥35	131	35	0.12 (0.08–0.20)	2.73 (1.15–6.51)	0.023*
Education level	Diploma	40	61	1	1	
	1st degree	69	111	0.95 (0.58–1.56)	0.40(0.14–1.14)	0.085
	2nd degree	100	32	4.77 (2.71–8.37)	0.97 (0.23–4.02)	0.961
Monthly income (dollar)	110.74–259.16	68	142	1	1	
	259.17–598.00	141	62	4.75 (3.13–7.20)	1.81 (0.60–5.50)	0.293
Marital status	Not married	53	126	1	1	
	Married	156	78	4.76 (3.12–7.24)	1.27 (0.59–2.76)	0.545
Experience in the bank (years)	<2	28	43	1	1	
	2–5	59	135	0.67 (0.38–1.18)	0.26 (0.10–0.71)	0.008*
	>5	122	26	7.21 (3.81–13.63)	0.74 (0.21–2.62)	0.636
Position as cashier (days/week)	0–4	58	72	1	1	
	5–6	151	132	1.42 (0.94–2.16)	1.60 (0.70–3.66)	0.269
Family size (persons)	<5	91	154	1	1	0.319
	≥5	118	50	3.99 (2.62–6.08)	0.67 (0.31–1.46)	
Have children	No	74	122	1	1	
	Yes	135	85	2.71 (1.82–4.04)	0.67 (0.32–1.39)	0.284
Have family members >65 years old in household	No	160	173	1	1	
	Yes	49	31	1.71 (1.04–2.81)	1.17 (0.51–2.69)	0.719
Presence of poster showing COVID-19 preventive measures at work	No	152	170	1	1	
	Yes	57	34	1.88 (1.16–3.02)	1.75 (0.76–4.02)	0.189
Chronic illness	No	156	177	1	1	
	Yes	53	27	2.23 (1.34–3.71)	2.24 (0.96–5.22)	0.061
Received training on COVID-19	No	134	175	1	1	
	Yes	75	29	3.38 (2.08–5.48)	0.48 (0.19–1.22)	0.121
Have health information on COVID-19	No	19	76	1	1	
	Yes	190	128	5.94 (3.42–10.30)	2.20 (0.85–5.70)	0.104
Knowledge about COVID-19	No	10	53	1	1	
	Yes	199	151	6.99 (3.44–14.2)	1.24 (0.45–3.43)	0.682
Attitude toward COVID-19 prevention	Negative	26	179	1	1	
	Positive	183	25	50.4 (28.0–90.6)	35.4(16.20–77.43)	<0.001*

AOR, adjusted odds ratio; COR, crude odds ratio; CI, confidence interval; 1, reference category. *Significant association.

## Discussion

In this study 84.7% of bank workers had good knowledge about COVID-19. Furthermore, 50.4% had a positive attitude towards taking COVID-19 precautions. This study also shows that 50.6% of bank workers had good practice of COVID-19 preventive measures.

Good knowledge about COVID-19 among bank workers in this study was 84.7% (95% CI: 81.1–88.1), the result is similar to the finding of a study among Tanzanian residents which was 84.4% (30). On the other hand, it was higher than studies done in Jimma 41.3% (41), Dessie and Kombolcha City 45.89% (43), Addis Ababa 37.2% (10), south Gondar Zone hospitals 69.3% (36), Nepal 76% (44), Hong Kong which was very low (45), Bangladesh 48.3% (31), and Syrian residents 60% (46). The high result in this study may be due to the study setting being an institution (bank) where more workers are expected to have good knowledge; it may also be due to variations in socio-demographic characteristics of the study participants. But this study’s result was lower than found by study among hospital visitors at Ataye district hospital, in Ethiopia 95.1% (47), and also compared to a study of the general population in Indonesia where the level of knowledge was positive (48), a study of most Chinese residents (29) and a majority of participants in a study in Saudi Arabia (49). This may be due to difference in study community or setting from which sample was taken.

Bank workers who had a positive attitude towards taking COVID-19 precautions were 8.89 times more likely to have good knowledge about COVID-19 from the present study. Similar results were found by studies conducted in Addis Ababa (10), and China (29). The reason why having a positive attitude contributes to have a strong knowledge might be that individuals who have a favorable attitude toward learning about COVID-19 are willing to read and gather information, and therefore their knowledge level rises. It might also be that a person who sees the risk seeks to learn about illnesses and how to protect themselves.

Good attitude towards taking precautions against COVID-19 among bank workers in this study was 50.4% (95% CI: 45.5–55.0). It is similar to study in Nepal at 54.7% (44). Similarity of result in these studies may be due to similarity in study settings and participants. This result in the current study is lower than of a study from Syria, which showed the overall attitudes score were higher at 63.5% (46), and also from Bangladesh 62.3% (31), south Gondar Zone hospitals 62.6% (36), Indonesia where the attitude of all participants was positive (48) and Addis Ababa where it was 60.7% (10). The reason for the more negative attitude found in this study may be that participants’ perception of the danger of the disease is low because of relatively low disease effects reported in our study area compared to other study settings or the disease effects not being clearly known by the current study’s participants. On the other hand, the attitude found in this study was higher than found by a study in Saudi Arabia where the mean score for attitude was 28.23% (49). This might be due to differences in study units.

Respondents with greater or equal to 35 years age were 2.46 times more likely to have a positive attitude towards taking COVID-19 precaution. A similar significant association was found by studies done in Nepal (44) and Bangladesh (31). This may be due to the fact that older individuals know they are more vulnerable to getting serious COVID-19 symptoms compared to younger people, and therefore have good attitude toward applying preventive measures to protect themselves. Furthermore, being married and having children were significantly associated with having a positive attitude towards taking COVID-19 precautions. The reason for this may be that these individuals were responsible for the care of others in their household in contrast to those who had only to care for themselves.

In this study bank workers who got health information about COVID-19 were 3.81 times more likely to have a positive attitude towards taking COVID-19 precautions. This finding is similar to that of a study in China (29). This may be because those who had information about the disease understood why and how to apply preventive. The present study found that bank workers having good knowledge were 10.22 times more likely to have a positive attitude towards taking COVID-19 precautions, a result similar to that of a study conducted in Addis Ababa (10). The reason for a positive attitude contributing to having good knowledge may be that those having a positive attitude toward knowing about COVID-19 are ready to read and get information, which in turn increases their knowledge level. In addition, knowledge may affect a person’s perception of the risks of getting the disease.

Practice of COVID-19 preventive measures among bank workers in this study was 50.6% (95% CI: 45.8–55.0). This result is similar to that of a study conducted in south Gondar Zone hospitals at 49.3% (36). This result was lower than that of a study from Indonesia, where the level of good practices was high (48), and in Addis Ababa at 59.8% (10), among frontline healthcare workers in Nepal at 78.9% (44), a study in Hong Kong where participants often implemented recommended disease-preventive measures such as maintaining social distance (88.1%) and wearing masks in public (94.3%) (45), among Syrians at 73.75% (46), a Bangladesh study where 55.1% had more frequent practices regarding COVID-19 (31), and good practices found by a study done in Saudi Arabia (29). On the other hand, the practice of prevention measures in this study was higher than found by a study done in Ataye district hospital 14.62% (47). The differences in practice level of participants in this study may be due to difference in study period, especially where there may have been government enforcement at the beginning of the disease outbreak.

In this study, a female was 2.56 times more likely to have a good practice than a male. Similar results were found from studies in Jimma (41), Bangladesh (31), China (29), Hong Kong (45), Saudi Arabia (49), and Syria (46). The reason for this may be that women worry more than men about COVID-19 disease for themselves, their families and individuals with whom they have contact.

This study shows that those 35 years of age or over were 2.73 times more likely to have good practices. Older age was associated with prevention practice in studies done in Ethiopia (47), Bangladesh (31), and Syria (46). Since older individuals are highly vulnerable to getting serious COVID-19 compared to younger people, they may be motivated to practice good COVID-19 preventive measures. Those bank workers having 2–5 years’ work experience were 0.26 times less likely to have good practice than those who had less than 2 years’ experience. This may be due to those having less work experience being younger than those with longer experience; older age was significant in this study.

Furthermore, those who had a positive attitude were significantly associated with practice of COVID-19 preventive measures. Attitude and self-efficacy to control COVID-19 were factors for COVID-19 preventive measures in studies in Jimma (41), Bangladesh (31) and Addis Ababa (10). Participants who perceived a lower risk of being infected and lower self-efficacy were less likely to implement preventive measures in Hong Kong (45). This perception of risk of getting the disease may be a factor associated with applying COVID-19 preventive measures since a person who perceives a risk may try to use preventive techniques for self-protection.

### Limitations of the study

Limitations of this study include using community-level and other institution studies for discussion as a result of scarcity of COVID-19-related studies on KAP of bank workers, the self-administration of the questionnaire for the sake of COVID-19 prevention and allowance of only a short time for workers to respond, which might have biased the self-reported data. Despite these limitations, this study can provide appropriate information about KAP level of bank workers in Dessie City.

### Practical implication of the study for practice/policy makers

For effective planning and implementation of preventive measures in this population, it is crucial to understand the KAP of Dessie City bank workers during the COVID-19 outbreak. Based on the results of this study, it is recommended that an institution-based health education program about COVID-19 be established as a necessary step to control the disease and that policy makers use appropriate interventions to control COVID-19 and improve the situation in future outbreaks by increasing bank workers’ knowledge, attitude and practice status.

## Conclusion

Our findings revealed good knowledge, but considerably negative attitude and poor practice towards COVID-19 among bank workers in Dessie City. The factor significantly associated with good knowledge about COVID-19 was a positive attitude towards taking COVID-19 precautions. Factors significantly associated with positive attitude towards COVID-19 precautions includes age being 35 years or over, and marital status Being female, and having 2–5 years’ work experience were among factors significantly associated with good preventive practice against COVID-19. It is recommended that bank manager’s work together with concerned bodies to improve KAP level of bank workers and that health decision makers develop updated guidance for bank workers. This can be by giving health education program and information dissemination to improve bank workers’ COVID-19 KAP level, including appropriate strategies by policy makers and bank managers to develop effective interventions to control COVID-19 transmission in banks.

## Data availability statement

The original contributions presented in the study are included in the article/supplementary material, further inquiries can be directed to the corresponding authors.

## Author contributions

SH and MA contributed to the conceptualizations of the study, methodology, validation, and statistical analysis, coordinated the data collection, drafted the original manuscript, and performed the statistical analysis and supervision. MA edited the manuscript. All authors read and approved the manuscript.

## Abbreviations

AOR: Adjusted Odds Ratio
CI: Confidence Interval
COR: Crude Odds Ratio
COVID-19: Coronavirus disease 2019
KAP: Knowledge Attitude and Practice
WHO: World Health Organization
